This article has been retracted.

# Effects of Deep Hyperthermia Combined with Intraperitoneal Chemotherapy on Liver-Kidney Function, Immune Function, and Long-Term Survival in Patients with Abdominal Metastases

**DOI:** 10.1155/2023/5878402

**Published:** 2023-04-21

**Authors:** Yan Zhang, Xiaomin Lu, Haoming Ji, Liangfeng Zheng, Guodong Chen, Ye Qian

**Affiliations:** ^1^Department of Oncology, Affiliated Hai'an Hospital of Nantong University, Nantong City, Jiangsu 226600, China; ^2^Cancer Central Laboratory, Affiliated Hai'an Hospital of Nantong University, Nantong City, Jiangsu 226600, China

## Abstract

**Objectives:**

To analyze the effects of deep hyperthermia combined with intraperitoneal chemotherapy on liver-kidney function, immune function, and long-term survival in patients with abdominal metastases.

**Methods:**

A total of 88 patients with abdominal metastases confirmed in the hospital were enrolled as the research objects between August 2018 and August 2021. They were randomly divided into control group (*n* = 44) and observation group (*n* = 44). The control group was treated with intraperitoneal chemotherapy, while observation group was additionally treated with deep hyperthermia. The general clinical data of patients were recorded. The short-term and long-term curative effects were evaluated. The occurrence of side effects in both groups was recorded. Before and after treatment, levels of alanine transaminase (ALT) and aspartate transaminase (AST) were detected by full-automatic biochemical analyzer. The level of blood urea nitrogen (BUN) was detected by the urease electrode method. The level of serum creatinine (Scr) was detected by the picric acid method. The levels of CD_3_^+^, CD_4_^+^, CD_8_^+^, and NK cells were detected by BD FACSCalibur flow cytometer.

**Results:**

There was no significant difference in clinical data between the two groups (*P* > 0.05). In the observation group, ORR was significantly higher than that in the control group (54.55% *vs* 29.55%) (*P* < 0.05), OS was significantly longer than that in the control group (*P* < 0.05), and median survival time and mPFS were longer than those in the control group. After treatment, the levels of ALT, AST, BUN, and Scr were significantly increased in the control group (*P* < 0.05), but there was no significant difference in peripheral blood CD_3_^+^, CD_4_^+^, and CD_4_^+^/CD_8_^+^ ratio or count of NK cells before and after treatment (*P* > 0.05). Before and after treatment, there was no significant difference in the levels of ALT, AST, BUN, and Scr in the observation group (*P* > 0.05). After treatment, peripheral blood CD_3_^+^, CD_4_^+^, and CD_4_^+^/CD_8_^+^ ratio and count of NK cells were all increased in the observation group, significantly higher than those in the control group (*P* < 0.05). The incidence of chemotherapy side effects in the observation group was significantly lower than that in the control group (*P* < 0.05).

**Conclusion:**

The short-term and long-term curative effects of deep hyperthermia combined with intraperitoneal chemotherapy are good on patients with intraperitoneal metastases, with less damage to liver-kidney function. It is beneficial to enhance immune function of patients, with mild side effects.

## 1. Introduction

Abdominal metastasis refers to the fact that solid malignant tumors in other parts of the body have invaded the abdomen, usually indicating that the patient has entered the advanced stage of cancer and has lost the surgical indications and no chance of radical cure, and the survival rate of patients can only be improved by chemotherapy and radiotherapy [1–3]. Patients with abdominal metastasis of tumor have complicated condition, rapid changes, poor prognosis, and difficult clinical treatment. In addition, they often have severe abdominal pain, abdominal distension, and other accompanying symptoms [4, 5]. Tumor chemotherapy has developed rapidly and achieved outstanding results in various tumor treatment fields. For patients with intraperitoneal metastases with severe ascites and other conditions, intraperitoneal chemotherapy is one of the best choices for prolonging survival. However, chemotherapy itself is accompanied by many complications. At the same time, due to drug resistance and more serious side effects, patients often have to stop chemotherapy after a period of treatment [6–8]. Tumor hyperthermia is an important part of the tumor treatment sector. Relying on the rapid development of medical technology in recent years, the clinical application of hyperthermia technology is becoming more and more mature, and the treatment effect can be improved by combining with chemotherapy. Deep hyperthermia, as one of the comprehensive therapies for tumors, combines chemotherapy with hyperthermia to scientifically and reasonably formulate clinical treatment plans and exert the synergistic effects of hyperthermia and chemotherapy, in order to improve the survival rate, alleviate the pain and improve the quality of life. Thermal therapy can expand blood vessels of tumor tissues, accelerate blood circulation, increase the concentration of chemotherapeutic drugs in tumor tissues, and promote the drugs to approach target cells [9, 10]. Meanwhile, thermal therapy can change cell permeability, increase the entry of chemotherapeutic drugs into cells, and enhance chemotherapy reaction [11]. This study investigated the effects of deep hyperthermia combined with intraperitoneal chemotherapy on liver and kidney function, immune function and long-term survival in patients with intra-abdominal metastases, in order to provide more possibilities for the treatment of advanced clinical malignant tumors. The report is as follows:

## 2. Materials and Methods

### 2.1. General Information

A total of 88 patients diagnosed with abdominal metastases in our hospital from August 2018 to August 2021 were selected as the research objects and randomly divided into the control group (*n* = 44) and the observation group (*n* = 44). Inclusion criteria: ① Meet the diagnostic criteria of various malignant tumors, confirmed by pathological diagnosis; ②Imaging examination showed that the tumor had abdominal metastasis; ③ Estimated lifetime is greater than or equal to 3 months; ④ No prior chemotherapy and immunotherapy; ⑤ Patients have good tolerance to deep hyperthermia and can cooperate with experimental research. Exclusion criteria: ① Patients with metal implants or contraindications to hyperthermia in areas requiring deep hyperthermia.; ② Patients with abnormal coagulation function or grade 3 hematological toxicity; ③ Patients with poor mental state or cognitive impairment; ④ Less than one assessable lesion;

### 2.2. Treatment Methods

Routine blood, liver and kidney function, electrocardiogram, and other routine examinations were performed in both groups before treatment.

The control group was treated with intraperitoneal chemotherapy. The patients were instructed to take a supine position for paracentesis, and infused with 150 ml of normal saline at 40°C. After successful infusion, cisplatin and mitomycin were added to about 2000 ml of normal saline to prepare chemotherapy drugs. Good chemotherapy drugs are injected into the abdominal cavity through a drainage tube, Make the drug directly interact with residual cancer cells in the abdominal cavity. During the treatment process, the abdominal cavity temperature is maintained at 40–42°C. At the same time, sodium sulfide sulfate is intravenously infused to reduce renal toxicity. After the infusion is completed, the patient should be changed every 15 minutes. Distributed to the tumor surface to achieve therapeutic effect, treatment was once every 1 week for a total of 4 weeks.

The observation group was treated with deep hyperthermia combined with intraperitoneal chemotherapy, and the intraperitoneal chemotherapy was the same as the control group. The patient's anatomical location of the tumor was confirmed by imaging diagnosis, and the EHY-200 ion radiofrequency deep hyperthermia machine was used for deep hyperthermia. According to the treatment needs, the patient was placed on the treatment water bed in the appropriate position, and the appropriate probe was placed in the well-covered tumor area and the abdominal cavity. Deep hyperthermia was performed about 30 minutes after chemotherapy, 1 hour each time, 3 times a week, for a total of 4 weeks.

### 2.3. Observation Indicators

#### 2.3.1. Efficacy Criteria [12]

After the treatment, the patients in the control group and the observation group underwent imaging examination to observe the clinical effect and evaluate the short-term effect of the patients. Complete remission (CR): Imaging results show that abdominal metastases and ascites have completely disappeared and can be maintained for more than 4 weeks; Partial remission (PR): The intraabdominal metastatic tumor was reduced by 50%, the ascites disappeared, and it was maintained for more than 4 weeks; Stable disease (SD): The volume of intra-abdominal metastases has decreased by less than 25% or increased by less than 25%, and no new lesions have been found to metastasize; Progressive disease (PD): The volume of metastatic tumor in abdominal cavity increased by more than 25% or a new tumor appeared.

Objective remission rate (ORR) = (CR + PR)/total number of cases × 100%.

#### 2.3.2. Liver and Kidney Function

*(1) Liver Function Indicators*. Before and after treatment, the levels of Alanine Transaminase (ALT) and Aspartate Transaminase (AST) were detected by Beckman LX-20 automatic enzyme immunoassay biochemical analyzer.

*(2) Kidney Function Indicators*. Before and after treatment, 3 mL of venous blood was drawn from all patients on an empty stomach in the early morning, placed in blood collection tubes without anticoagulant, centrifuged to separate serum, and stored in a −20°C refrigerator for testing. Blood urea nitrogen (BUN) level and serum creatinine (Scr) level were detected by the urease electrode method.

#### 2.3.3. Immune Function

Before and after treatment, 5 mL of fasting venous blood was collected from the two groups of patients in the morning, anticoagulated, and centrifuged to get the supernatant, which was stored in a −40°C refrigerator for testing. Reagents were purchased from BD Company.

#### 2.3.4. Lifetime

The patients were followed up for 1–48 months by means of telephone follow-up, and the follow-up deadline was August 2022. Telephone follow-up was conducted for 1–48 months with a follow-up deadline of August 2022. The death of the patient due to tumor was considered as the follow-up endpoint. The median survival time, overall survival (OS), and median progression-free survival (mPFS) of patients were recorded.

#### 2.3.5. Case Elimination Criteria

Patients with telephone loss; patients who die from non-neoplastic progression; patients who withdrew from the study due to their own volition. Finally, a total of 5 patients were lost to follow-up during the follow-up period.

#### 2.3.6. Safety Evaluation

The occurrence of toxic and side effects of chemotherapy in the two groups of patients during treatment, including nausea and vomiting, thrombocytopenia, leukopenia, diarrhea, bone marrow suppression, and hepatotoxicity, were recorded.

### 2.4. Statistical Processing

SPSS 21.0 software was used to analyze the obtained data, and the measured data conforming to the normal distribution is expressed by the ($\bar{x}$  ± *s*), and the *t*-test was used to analyze the differences of parameter between the two groups; The enumeration data were expressed as rate (%), and the *χ*^2^ test was used to compare the categorical data; The survival curve was drawn by Kaplan-Meier (K-M) analysis, and the survival rate was compared by Log Rank *χ*^2^ test; *P* < 0.05 indicated statistical significance.

## 3. Results

### 3.1. Comparison of Clinical Data between the Two Groups of Patients

There was no significant difference in clinical data between the two groups (*P* > 0.05). As shown in Table 1.

### 3.2. Comparison of Short-Term Curative Effect between Two Groups of Patients

The ORR of the observation group was 58.54%, and the ORR of the control group was 30.95%. The ORR of the observation group was significantly higher than that of the control group (*P* < 0.05). As shown in Table 2.

### 3.3. Long-Term Survival Analysis of Two Groups of Patients

During the follow-up process, 5 cases were lost to follow-up, and the total sample size was 83 cases, including 3 cases in the control group and 2 cases in the observation group. The follow-up time was 1–48 months. The OS of the observation group was significantly longer than that of the control group (*P* < 0.05), and the median survival time and mPFS were longer than those of the control group. As shown in Figure 1 and Table 3.

### 3.4. Comparison of Liver and Kidney Function between the Two Groups before and after Treatment

After treatment, the levels of ALT, AST, BUN, and Scr in the control group were significantly increased compared with those before treatment (*P* < 0.05). Before and after treatment, there was no significant difference in the levels of ALT, AST, BUN, and Scr in the observation group (*P* < 0.05). As shown in Figure 2.

### 3.5. Comparison of Immune Function between the Two Groups before and after Treatment

After treatment, the peripheral blood CD_3_^+^ level, CD_4_^+^ level, and CD_4_^+^/CD_8_^+^ ratio and NK cell count in the observation group were all increased and were significantly higher than those in the control group (*P* < 0.05). Before and after treatment, there were no significant differences in peripheral blood CD_3_^+^ level, CD_4_^+^ level, and CD_4_^+^/CD_8_^+^ ratio and NK cell count in the control group (*P* > 0.05). As shown in Figure 3.

### 3.6. Comparison of Toxic and Side Effects of Chemotherapy in the Two Groups of Patients

After treatment, both groups of patients developed chemotherapy toxicity, but the reaction was mild. The incidence of chemotherapy toxicity and side effects such as nausea and vomiting, thrombocytopenia, leukopenia, diarrhea, bone marrow suppression, and hepatotoxicity in the observation group was significantly lower than that in the control group (*P* < 0.05). As shown in Table 4.

## 4. Discussions

Abdominal metastasis is a form of metastasis that occurs when malignant tumors develop to an advanced stage, which marks the development of solid tumors from local to systemic metastasis. At present, the diagnosis and treatment methods for intraabdominal metastases are not perfect, and the adverse effects of intraabdominal metastases on the survival of patients have not been completely eliminated [13–15]. The two-in-one comprehensive treatment model combining hyperthermia and chemotherapy is a research hotspot recently. After years of clinical verification, it has been shown that this treatment plan is a comprehensive measure with definite curative effect and no strong toxic and side effects, and has effectively solved a number of clinical malignant tumors [16–18]. The results of this study showed that the ORR of the patients in the observation group was significantly higher than that in the control group, suggesting that deep hyperthermia combined with intraperitoneal chemotherapy had a higher clinical remission rate for intraperitoneal metastases and showed a more impressive clinical effect. This may be because the chemotherapeutic drugs are directly injected into the abdominal cavity, which avoids the effect of the “peritoneal-plasma barrier” on drug absorption, ensures the amount and concentration of chemotherapeutic drugs entering the abdominal cavity, and makes them in direct contact with the tumor. The synergistic effect of deep hyperthermia increases the sensitivity of tumors to chemotherapy and can effectively kill free cancer cells and micrometastases in the abdominal cavity [19, 20]. In addition to directly inhibiting the growth of malignant tumor cells and accelerating the process of cancer cell apoptosis, deep hyperthermia can also stimulate the body's immune system by synthesizing heat shock proteins, improve the body's immunity, and help resist malignant tumors [21, 22]. Long-term follow-up investigation of patients in two groups showed that OS of the observation group was significantly superior to that of the control group, and the median survival time and mPFS of the observation group were also longer than those of the control group, indicating that deep hyperthermia combined with intraperitoneal chemotherapy could facilitate the long-term survival, improve the long-term survival rate, extend the progression-free survival time, and improve the quality of life of patients during the anticancer process.

The results of this study showed that the levels of ALT, AST, BUN, and Scr in the control group increased significantly after treatment, while there was no significant difference in the indicators in the observation group, indicating that the liver and kidney function of the patients decreased after only intraperitoneal chemotherapy. After combined with deep hyperthermia, liver and kidney functions were not significantly damaged compared with those before treatment. Although deep hyperthermia did have negative effects on liver and kidney functions, these effects were mostly transient pathological changes and would not cause serious liver and kidney disease [23]. The results of this study also showed that there were no statistical changes in CD3+ level, CD4+ level, and CD4+/CD8+ ratio and NK cell count in the control group before and after treatment. The abovementioned indicators in the observation group were all increased after treatment as compared with those before treatment, suggesting that the immune function of patients was significantly improved after deep hyperthermia combined with intraperitoneal chemotherapy. The incidence of toxic and side effects of chemotherapy in the two groups after treatment was observed, and it was found that the incidence of toxic and side effects of chemotherapy in the observation group was significantly lower than that in the control group, and the adverse reactions were mild, indicating that the deep hyperthermia combined with chemotherapy had higher safety and made patients more easily adapt to chemotherapy. The reason why deep hyperthermia can make patients tolerate chemotherapy may be that thermodynamic effect improves the hemodynamics of liver and kidney tissues, increases the blood flow of the body and accelerates metabolism, thus reducing the toxic damage of liver and kidney during chemotherapy [24, 25].

In conclusion, deep hyperthermia combined with intraperitoneal chemotherapy can improve the clinical remission rate of patients with abdominal metastases, and enable patients to achieve short-term and long-term survival benefits, which might be due to the fact that deep hyperthermia reduced the toxicity of chemotherapy to the liver and kidney and improved the immune function of the patients.

## Figures and Tables

**Figure 1:** OS of the two groups of patients.

**Figure 2:** Comparison of liver and kidney function before and after treatment in two groups of patients. Note: compared with before treatment, ^*∗*^*P* < 0.05.

**Figure 3:** Comparison of immune function between the two groups before and after treatment. Note: compared with before treatment, ^*∗*^*P* < 0.05.

**Table 1:** Comparison of clinical data of the two groups of patients (*n*, %).

Indexes	Control group (*n* = 44)	Observation group (*n* = 44)	*t/χ* ^*2*^	*P*
Gender			0.741	0.389
Male	23	27		
Female	21	17		
Age (year)	59.05 ± 8.72	60.31 ± 8.54	0.653	0.516
Course of disease (d)	9.85 ± 2.16	10.32 ± 2.47	0.906	0.368
ECOG scale (score)			1.216	0.544
1	12	9		
2	25	30		
3	7	5		
Primary tumor site			1.687	0.975
Gastrointestinal	13	15		
Esophagus	2	3		
Pancreas	8	6		
Liver	8	9		
Gallbladder	5	5		
Ovary	3	1		
Breast	2	2		
Cervix	3	3		

**Table 2:** Comparison of short-term curative effect between two groups of patients (*n* = 44, %).

Group	CR	PR	SD	PD	ORR (%)
Control group	4	20	15	2	24/41
Observation group	1	12	22	7	13/42
*χ* ^*2*^					5.643
*P*					0.018

**Table 3:** Survival analysis of the two groups of patients.

Group	Median survival (months)	OS (%)	mPFS (months)
Control group (*n* = 41)	20.21	5/41 (12.20)	6.35
Observation group (*n* = 42)	28.93	11/42 (26.19)	10.47
Log rank *χ*^2^	—	5.776	—
*P*	—	0.016	—

**Table 4:** Comparison of toxic and side effects of chemotherapy in two groups of patients (*n* = 44, %).

Group	Nausea and vomiting	Thrombocytopenia	Leukopenia	Diarrhea	Bone marrow suppression	Hepatotoxicity
Control group	35	40	35	29	33	19
Observation group	26	33	20	17	21	8
*χ* ^*2*^	4.328	3.938	10.909	6.559	6.902	6.465
*P*	0.037	0.047	0.001	0.010	0.009	0.011

## Data Availability

The raw data supporting the findings of this article will be available from the corresponding author upon request.
